The article "A Smoothed Matrix Multivariate Elliptical Distribution-Based Projection Method for Feature Extraction" was published in 2022. Journal: Comput Intell Neurosci.

# A Smoothed Matrix Multivariate Elliptical Distribution-Based Projection Method for Feature Extraction

**DOI:** 10.1155/2022/2551137

**Published:** 2022-09-30

**Authors:** Hong Qiu, Renfang Wang, Dechao Sun, Xinwei Liu, Liang Zhang, Yunpeng Liu

**Affiliations:** ^1^College of Big Data and Software Engineering, Zhejiang Wanli University, Ningbo 315100, China; ^2^College of Digital Technology and Engineering, Ningbo University of Finance and Economics, Ningbo 315175, China; ^3^College of International Exchange, Ningbo University of Technology, Ningbo 315211, China

## Abstract

Big data has the traits such as “the curse of dimensionality,” high storage cost, and heavy computation burden. Self-representation-based feature extraction methods cannot effectively deal with the image-level structural noise in the data, so how to character a better relationship of reconstruction representation is very important. Recently, sparse representation with smoothed matrix multivariate elliptical distribution (SMED) using structural information to handle low-rank error images caused by illumination or occlusion has been proposed. Based on SMED, we present a new method named SMEDP for feature extraction. SMEDP firstly utilizes SMED to automatically construct an adjacency graph and then obtains an optimal projection matrix by maximizing the ratio of the local scatter matrix and the total scatter matrix in the PCA subspace. Experiments on the COIL-20 object database, ORL face database, and CMU PIE face database prove that SMEDP works well and can achieve considerable visual and recognition performance than the relevant methods.

## 1. Introduction

Big data analytics as the premise and the foundation of artificial intelligence can easily cause the problem of “curse of dimensionality” [1], high storage cost, and heavy computation burden [2]. How to deal with such high-dimensional data is always a vital issue in many applications, including machine intelligence, data mining, pattern recognition, and image processing [3–5]. Feature extraction can effectively solve the above problems by reducing the size of a data set while preserving relevant information. Thus, it has become a research hotspot [6–8].

Principle component analysis (PCA) [9]and linear discriminant analysis (LDA) [10] are two commonly used linear feature extraction methods. The former projects the high-dimensional data by maximizing the variance while the latter maximizing the ratio of the between-class scatter matrix and the within-class scatter matrix. Although they are simple and effective for some practical applications, they may fail to discover the underlying manifold structures of the observed data that are nonlinear.

The article "A Smoothed Matrix Multivariate Elliptical Distribution-Based Projection Method for Feature Extraction" was published in 2022. Journal: Comput Intell Neurosci.

To discover the intrinsic low-dimensional embedding of the observed data, researchers developed many manifold learning methods. Isometric feature mapping (ISOMAP) [11], Laplacian eigenmaps (LE) [12], and locally linear embedding (LLE) [13] are the most representative methods. They try to preserve the intrinsic geometrical distribution of the high-dimensional data. ISOMAP takes the pairwise geodesic distance between samples as the feature of manifold structure, and LE builds the neighborhood information graph to maintain the neighborhood relationships among the samples, while LLE believes that local relations characterize the manifold structure of data. Although they are excellent in some respects, there are still some problems, such as sensitivity to noise and “out-of-sample” problem. Thus, as improvement methods, neighborhood preserving embedding (NPE) [14], locality preserving projections (LPP) [15], and so on have been proposed. NPE and LPP are the linearized versions of LE and LLE, and they focus on the local information of the data and linearize the nonlinear structure to handle the “out-of-sample” problem. But apparently, the *k*-nearest graph or the *ε*-ball graph they use is very sensitive to parameter settings and noise interference [16].

Numerous researchers study it constantly to solve these problems. They found that the methods mentioned above can be unified with a graph embedding framework [17]. It is critical to construct adjacency graphs in this framework, which can effectively reveal the essential structure of the data. More recently, sparse representation (SR)-based methods are adopted to automatically construct adjacency graphs, since it has the advantages of sparsity, robustness to noise, and datum-adaptive neighborhood. For instance, Qiao et al. [18] developed a sparsity preserving projections (SPP) by using a modified SR-based classification (SRC) [19] to automatically build the graph. And then, the projections are obtained such that the sparse reconstructive relationship of the data can be best preserved. But it is a time-consuming process since SPP aims to solve the L_1_-norm optimization problem. Therefore, Yang et al. [20] solved the L_2_-norm optimization problem instead of the L_1_-norm optimization to reduce the running time, and proposed a collaborative representation-based projection (CRP). It benefits from the collaborative representation classifier (CRC) [21] and can obtain a comparable result with SPP. Note that both SPP and CRP choose their neighborhood automatically and contain natural discriminating information, hence can be more practical than some manifold learning methods.

The limitations that still exist though SPP and CRP work well in some applications. First, they are all vector-based methods. That means they need to stretch the image matrix into a vector in advance, which will ignore the spatial structural information of the data. Second, for many error images caused by illumination variations or occlusions, the assumption of independence of error variables may not be appropriate in some practical situations. Many SR works attempt to handle the above problems. Yang et al. [22] and Xu et al. [23] studied the illumination variations and occlusions caused error images and observed that the structure of error variables is low rank or approximately low rank [24]. They pointed out that low-rank constraints can be used to describe the structure noise, whereas it is NP-hard in solving the rank minimization problem [25]. A general way to address such an issue is to substitute the rank function with some tractable surrogate.

The article "A Smoothed Matrix Multivariate Elliptical Distribution-Based Projection Method for Feature Extraction" was published in 2022. Journal: Comput Intell Neurosci.

To this end, Yang et al. utilized nuclear norm to characterize the illumination variations and occlusions caused error images and developed a nuclear norm-based matrix regression model (NMR) [22]. Based on NMR, Yang et al. [26] explored NMR to construct the graph and gave a NMR-based projection (NMRP). NMRP has shown its promise in feature extraction. Qian et al. [27] integrated error detection and error support into one model and provided a robust nuclear norm regularized regression (RNR). Xie et al. [28] described the structural noise and the mixed noise by the robust nuclear norm and proposed a novel robust matrix regression (RMR). Significantly, these methods all assumed that each pixel of noise follows Gaussian or Laplacian distribution independently, which is not flexible for practical application. Therefore, some researchers are devoted to the study of low-rank representation (LRR) [29]. Fang et al. [30] improved the latent low-rank representation (LatLRR) [31], which is an excellent LRR-based feature extraction method. They proposed an approximate low-rank projection learning (ALP) and an extended ALPL (EALPL) to learn an optimal projection that can extract more discriminant features than LatLRR. Then, combining with rigid regression, they extended LatLRR to the supervised scenario and proposed a supervised ALPL (SALPL). Zhang et al. [32] introduced orthogonal matrix, row sparsity constraint on the projection matrix, and weighted truncated Schatten p-norm (WTSN) [32] to improve the robustness of the LRR model. However, these methods cannot handle the “out-of-sample” problem.

Recently, Qiu et al. [33] used a matrix multivariate elliptical distribution to characterize the error image and developed a sparse representation with smoothed matrix multivariate elliptical distribution (SMED). Compared with Gaussian or Laplacian distribution, a matrix multivariate elliptical distribution is more suitable for describing the structure noise. Besides, it introduces regularization terms to smooth the objective function, which makes the model easily to get a globally optimal solution. In short, SMED considers both of the global structure and the local structure based on sparse and low-rank representation. Thus, in this paper, we plan to explore SMED to automatically construct an adjacency graph and then learn an optimal projection matrix in the PCA subspace. The proposed method is named a smoothed matrix multivariate elliptical distribution-based projections (SMEDP). Since the projection matrix can be got directly, SMEDP can solve the “out-of-sample” problem well.

The article "A Smoothed Matrix Multivariate Elliptical Distribution-Based Projection Method for Feature Extraction" was published in 2022. Journal: Comput Intell Neurosci.

Figure 1 is the flowchart of our method, and the major contributions of this paper include: (1) in order to avoid the adverse effects produced by neglecting structural information, we propose a method named SMEDP. SMEDP can learn an adaptive graph with a modified SMED. (2) A method of iteratively reweighted least squares is designed to obtain the globally optimal weight matrix, which can be used to calculate the final projection matrix. (3) Comprehensive experiments have been carried out to indicate the superiority of SMEDP when compared with several relevant methods.

The rest of the paper is organized as follows.  Section 2 gives a brief review of SMED.  Section 3 introduces the SMEDP for feature extraction in detail. In Section 4, extensive experiments on three databases are presented to demonstrate the effectiveness of SMEDP.  Section 5 draws the conclusions and gives the prospect of the future work.

## 2. SMED

The idea of SR-based methods is to derive a series of appropriate representation coefficients. In the following, we give an overview of SMED [33].

Given a dataset of *n* training image matrices {**X**_1_^1^, **X**_2_^1^,…, **X**_*n*1_^1^, **X**_1_^2^, **X**_2_^2^,…, **X**_*n*2_^2^,…, **X**_1_^*C*^, **X**_2_^*C*^,…, **X**_*nC*_^*C*^}∈*R*^*p*^^×^^*q*^ and an image matrix **Y** ∈ *R*^*p*×*q*^, we can represent **Y** linearly using training image matrices, that is,

(1) $$\begin{array}{c} Y=X_{1}^{1}\alpha_{1}+X_{2}^{1}\alpha_{2}+,\ldots ,+X_{n1}^{1}\alpha_{n1}\\ +,\ldots ,+X_{1}^{C}\alpha_{n-nC}+,\ldots ,+X_{nC}^{C}\alpha_{n}+E, \end{array}$$

where **X**_*i*_^*c*^ represents the *i*-th training sample from the *c*th class, ***α*** = [*α*_1_, *α*_2_,…, *α*_*n*_]∈*R*^*n*^ is a vector of representation coefficients, and **E** is the structural noise.

To simplify the formula, linear mapping from *R*^*n*^ to *R*^*p*^ ^×^ ^*q*^ can be defined as follows:

(2) $$\begin{array}{c} X\left(\alpha \right)=X_{1}^{1}\alpha_{1}+X_{2}^{1}\alpha_{2}+,\ldots ,+X_{n1}^{1}\alpha_{n1}\\ +,\ldots ,+X_{1}^{C}\alpha_{n-nC}+,\ldots ,+X_{nC}^{C}\alpha_{n}. \end{array}$$

Then, (1) becomes

(3) $$\begin{array}{c} Y=X\left(\alpha \right)+E, \end{array}$$

(3) is a matrix variate-based linear model. Qiu et al. [33] have studied the error image and found that the correlations between pixels in **E** can be effectively alleviated by the proposed matrix multivariate elliptical distribution. Subsequently, a sparse representation with smoothed matrix multivariate elliptical distribution (SMED) model is developed to preserve the spatial information about the structural noise.

The article "A Smoothed Matrix Multivariate Elliptical Distribution-Based Projection Method for Feature Extraction" was published in 2022. Journal: Comput Intell Neurosci.

SMED assumes that **E** follows the matrix multivariate elliptical distribution and the set of representation coefficients follows the independent Gaussian distribution (*l* = 2) or Laplacian distribution (*l* = 1). Then, we have

(4) $$\begin{array}{c} \min_{\alpha }\xi \left(\alpha \right)=tr{\left(Y-X\left(\alpha \right)\right)}^{T}{\left(Y-X\left(\alpha \right)\right)}^{\frac{k}{2}}+\frac{1}{\beta }\overset{n}{\underset{i=1}{\sum }}{\left|\alpha \right|}_{l}^{l}\text{.} \end{array}$$

Based on the definitions of nuclear norm and *l*_*p*_-norm, (4) is equivalent to:

(5) $$\begin{array}{c} \min_{\alpha }\xi \left(\alpha \right)={\left\|Y-X\left(\alpha \right)\right\|}_{*}^{k}+\frac{1}{2}\lambda {\left\|\alpha \right\|}_{l}^{l}\text{,} \end{array}$$

where *λ* = 2/*β*, *k* > 0, and 0 < *l* ≤ 2. Since both two terms in (5) are nonsmooth, SMED introduces regularization terms to smooth them:

(6) $$\begin{array}{c} \min_{\alpha }\xi \left(\alpha ,\mu \right)={\left\|\left[\begin{array}{c} Y-X\left(\alpha \right)\\ \mu I \end{array}\right]\right\|}_{*}^{k}+\frac{1}{2}\lambda {\left\|\left[\begin{array}{c} \alpha \\ \mu 1 \end{array}\right]\right\|}_{l}^{l}\text{,} \end{array}$$

where *μ* is a penalty parameter, **I** ∈ *R*^*q*^ ^×^ ^*q*^ is an identity matrix, and **1**∈*R*^*n*^ is an all ones vector.

We obtain the optimal solution ***α***^*∗*^ by solving the (6), and the corresponding reconstruction error of the *i*-th class is defined as follows:

(7) $$\begin{array}{c} e_{i}\left(Y\right)={\left\|\hat{Y}-{\hat{Y}}_{i}\right\|}_{*}={\left\|X\left(\alpha^{*}\right)-X\delta_{i}\left(\alpha^{*}\right)\right\|}_{*}\text{,} \end{array}$$

where $\hat{Y}$ represents the reconstructed image of **Y**, ${\hat{Y}}_{i}$ means the reconstruction of **Y** in class *i*, and *δ*_*i*_(***α***^*∗*^) is a vector with only nonzero entries associated with the *i*-th class.

## 3. Algorithm Derivation of SMEDP

It is essential to construct adjacency graphs in graph-based feature extraction methods. Since SMED can better handle with variations of structural noise than several relevant methods, such as SRC and CRC, we explore SMED to automatically construct an adjacency graph and then seek to find a rule to get an optimal projection matrix. Subsequently, a method called smoothed matrix multivariate elliptical distribution-based projection method (SMEDP) is developed.

The article "A Smoothed Matrix Multivariate Elliptical Distribution-Based Projection Method for Feature Extraction" was published in 2022. Journal: Comput Intell Neurosci.

### 3.1. Constructing an Adjacency Graph

In this section, we will introduce how to construct an adjacency graph. Firstly, **X** = {**X**_*i*_^*c*^}∈*R*^*m*^ ^×^ ^*n*^, where *m* = *p* × *q* is adopted as the vertices of the graph. Secondly, smoothed matrix regression model based on the modified SMED is presented, and the method of iteratively reweighted least squares is used to solve the model to obtain the optimal weight vector ***α***_*i*_^*∗*^ for each **X**_*i*_(*i* = 1, 2,…, *n*). The edges of the graph are composed of a weight matrix ***α*** whose elements are ***α***_*i*_^*∗*^. Subsequently, Algorithm 1 describes each step of the procedure in detail.

The smoothed matrix regression model based on the modified SMED is defined as follows:

(8) $$\begin{array}{c} \alpha_{i}=argmin\left\{{\left\|\left[\begin{array}{c} X_{i}-X\left(\alpha_{i}\right)\\ \mu I \end{array}\right]\right\|}_{*}+\frac{1}{2}\lambda \left\|\left[\begin{array}{c} \alpha_{i}\\ \mu 1 \end{array}\right]\right\|\right\}, \end{array}$$

where the parameters *k* and *l* in (6) are set to 1, ***α***_*i*_ = [*α*_*i*1_,…, *α*_*i,i-*1_, 0, *α*_*i,i+*1_,…, *α*_*in*_]^T^, and the element *α*_*ij*_ (*i*≠*j*) in ***α***_*i*_ represents the contribution of each **X**_*i*_ to reconstruct**X**_*j*_.

Motivated by SMED, we provide details of using the method of iteratively reweighted least squares to solve Equation (8) [33], and it can be reformulated as follows:

(9) $$\begin{array}{c} \min_{\alpha_{i}}tr{\left({\left(X_{i}-X\left(\alpha_{i}\right)\right)}^{T}\left(X_{i}-X\left(\alpha_{i}\right)\right)+\mu^{2}I\right)}^{\frac{1}{2}}\\ +\frac{1}{2}\lambda {\left(\overset{n}{\underset{j=1}{\sum }}{\left|\alpha_{ij}\right|}^{2}+\mu^{2}\right)}^{\frac{1}{2}}\text{.} \end{array}$$

Let *γ*(***α***_*i*_) = tr((**X**_*i*_−**X**(***α***_*i*_))^T^(**X**_*i*_−**X**(***α***_*i*_)) + *μ*^2^**I**)^1/2^ and *δ*(***α***_*i*_)= (∑_*j*_ _=_ _1_^*n*^ |*α*_*ij*_|^2^ + *μ*^2^)^1/2^. Then, *ξ*(***α***_*i*_, *μ*) = *γ*(***α***_*i*_) + (*λ*/2)*δ*(***α***_*i*_). The derivative of *γ*(***α***_*i*_) is

(10) $$\begin{array}{c} \frac{\partial \gamma \left(\alpha_{i}\right)}{\partial \left(\alpha_{i}\right)}=\frac{\left(X^{T}X\alpha_{i}-X^{T}X_{i}\right)}{{\left({\left(X_{i}-X\left(\alpha_{i}\right)\right)}^{T}\left(X_{i}-X\left(\alpha_{i}\right)\right)+\mu^{2}I\right)}^{-1/2}}\\ ≜\left(X^{T}X\alpha_{i}-X^{T}X_{i}\right)R\text{,} \end{array}$$

where **R** = ((**X**_*i*_−**X**(***α***_*i*_))^T^(**X**_*i*_−**X**(***α***_*i*_)) +*μ*^2^**I**) ^−1/2^. The derivative of *δ* (***α***_*i*_) is as follows:

(11) $$\begin{array}{c} \frac{\partial \delta \left(\alpha_{i}\right)}{\partial \left(\alpha_{i}\right)}=\frac{\alpha_{i}}{{\left(\overset{n}{\underset{j=1}{\sum }}{\left|\alpha_{ij}\right|}^{2}+\mu^{2}\right)}^{-1/2}}≜\alpha_{i}T\text{,} \end{array}$$

where ***T***=(Σ_*j*_ _=_ _1_^*n*^|*α*_*ij*_|^2^ + *μ*^2^)^-1/2^.

The article "A Smoothed Matrix Multivariate Elliptical Distribution-Based Projection Method for Feature Extraction" was published in 2022. Journal: Comput Intell Neurosci.

With the derived *γ*(***α***_*i*_) and *δ* (***α***_*i*_), we get the derivative of *ξ*(***α***_*i*_, *μ*). By setting it to 0, we obtain that:

(12) $$\begin{array}{c} \frac{\partial \xi \left(\alpha_{i}\right)}{\partial \left(\alpha_{i}\right)}=\left(X^{T}X\alpha_{i}-X^{T}X_{i}\right)R+\frac{1}{2}\lambda l\alpha_{i}T=0\text{.} \end{array}$$

Or equivalently,

(13) $$\begin{array}{c} X^{T}X\alpha_{i}+\frac{1}{2}\lambda \alpha_{i}TR^{-1}=X^{T}X_{i}\text{.} \end{array}$$

As a well-known Sylvester equation, the computational complexity of (13) is *O*(*n*^3^) [34–36]. We can use MATLAB command lyap to get the weight matrix ***α*** **=** [***α***_1_, ***α***_2_,…, ***α***_*n*_]∈*R*^*n*×*n*^.

Algorithm 1 shows the detailed steps for solving ***α***.

### 3.2. Calculating the Projection Matrix

In this section, we will introduce how to calculate the projection matrix to improve classification performance. Firstly, we utilize PCA to reduce the dimensions of the raw data. Secondly, we seek to find an optimal projection matrix by maximizing the ratio of the local scatter matrix and the total scatter matrix in the PCA subspace. Subsequently, the final projection matrix is obtained based on the optimal projection matrix and the PCA-transformation matrix.

According to the ideas of CRP [20] and NMRP [26], the local scatter matrix is defined as follows:

(14) $$\begin{array}{c} \overset{n}{\underset{i=1}{\sum }}{\left\|P^{T}x_{i}-\overset{n}{\underset{j=1}{\sum }}\alpha_{ij}P^{T}x_{j}\right\|}^{2}=P^{T}X{\left(I-\alpha \right)}^{T}\left(I-\alpha \right)X^{T}P, \end{array}$$

where ***x***_*i*_ = Vec(**X**_*i*_) means the vector form of **X**_*i*_.

The total scatter matrix is expressed as follows:

(15) $$\begin{array}{c} \overset{n}{\underset{i=1}{\sum }}{\left\|P^{T}x_{i}-P^{T}\tilde{x}\right\|}^{2}=P^{T}\left(\overset{n}{\underset{i=1}{\sum }}\left(x_{i}-\tilde{x}\right){\left(x_{i}-\tilde{x}\right)}^{T}\right)P\\ =P^{T}\left(X-\tilde{X}\right){\left(X-\tilde{X}\right)}^{T}P\text{,} \end{array}$$

where $\tilde{x}$ is the mean vector of the training samples and the matrix $\tilde{X}$ is augmented by $\tilde{x}$.

The article "A Smoothed Matrix Multivariate Elliptical Distribution-Based Projection Method for Feature Extraction" was published in 2022. Journal: Comput Intell Neurosci.

So, the objective function of SMEDP is expressed as follows:

(16) $$\begin{array}{c} \min_{p}\frac{P^{T}X{\left(I-\alpha \right)}^{T}\left(I-\alpha \right)X^{T}P}{P^{T}\left(X-\tilde{X}\right){\left(X-\tilde{X}\right)}^{T}P}\text{.} \end{array}$$

Or equivalently,

(17) $$\begin{array}{c} \max_{p}\frac{P^{T}X\alpha_{\beta }X^{T}P}{P^{T}\left(X-\tilde{X}\right){\left(X-\tilde{X}\right)}^{T}P}\text{,} \end{array}$$

where ***α***_*β*_ **=** ***α*+*α***^T^**-*α***^T^***α***. Then, generalized eigenvector decomposition is adopted to solve Equation (17). The optimal projection matrix **P** can be calculated by

(18) $$\begin{array}{c} X\alpha_{\beta }X^{T}P=\lambda \left(X-\tilde{X}\right){\left(X-\tilde{X}\right)}^{T}P, \end{array}$$

where **P** = [***p***_1_, ***p***_2_,…, ***p***_*d*_] is the first *d* largest eigenvalues of Equation (18).

### 3.3. SMEDP

In this subsection, we summarize the details of SMEDP by Algorithm 2.

## 4. Experiments

We conduct experiments on COIL-20 object database, ORL face databases, and CMU PIE face databases to evaluate the performance of SMEDP. All the experiments are implemented in the same environment (CPU: Intel i7+ Lenovo, RAM: 8 GB, MATLAB: 2020b).

### 4.1. Experiments on COIL-20 Object Database

COIL-20 object database [37] contains 20 objects. For each object, 72 images are taken from different view directions. We use a subset of the COIL-20 for our experiments. This subset includes 50 images of 10 objects (each object has 5 images). All images were in grayscale and resized to 40 × 40 pixels. Figures 2 and 3 show some images.

We test the visual performance of SMEDP and compare it with the classical methods, that is, PCA; some manifold learning methods, that is, LLE, ISOMAP, and LPP; and SR-based methods, that is, SPP, CRP, and NMRP. The number of nearest neighbor point *k* in LEE, ISOMAP, and LPP is, respectively, set to 15, 20, and 20. We select Justin Romberg's l1qc_logbarrier to calculate L1-norm in SPP. Besides, the parameters in SPP, CRP, NMRP, and SMEDP are determined by grid search. In experiments, we start by using PCA to reduce the dimensions of the data to 70, and then adopt the above methods to convert the 70-dimensional representation to a 2-dimensional map.  Figure 4 shows the resulting map, where the color of a feature point in the scatterplot represents the class information of data.

From Figure 4, we can find that: (1) PCA confuses the projected data since it has a large variance. (2) LEE and ISOMAP fail to effectively separate data points, which are of different classes. Although they take into account the local structure of the data, the Euclidean distance measure or the geodesic distance measure cannot determine the real local structure. (3) The sparsity properties could enhance the visual performance, so the separation degree of SPP, CRP, and NMRP is better than LEE and ISOMAP. About SPP and CRP, CRP generates a smaller intraclass scatter in our experiment. This result demonstrates that it is the collaborative representation that plays an important role in the effectiveness of SRC. (4) The matrix-based methods usually surpass the vector-based methods (e.g., NMRP and our SMEDP method, which make use of the structural information outperform SPP). Notably, they enhance the performance of intraclass clustering. (5) NMRP can properly embed most classes, but some classes are still mixed. Its performance is inferior to CRP since the nuclear norm used in the matrix regression model is still a loose approximation to the natural rank constraint. (6) Due to the introduced regularization term in matrix regression model, our SMEDP method can achieve better results than others. Since SMEDP ignores the class label information, it also exists some overlapping phenomena among classes. We can try to absorb supervised information into the method to overcome the limitation further.

The article "A Smoothed Matrix Multivariate Elliptical Distribution-Based Projection Method for Feature Extraction" was published in 2022. Journal: Comput Intell Neurosci.

### 4.2. Experiments on ORL Face Database

ORL face database [38] consists 40 people. For each people, 400 images are taken from various illumination and facial expressions. All images were in grayscale and resized to 32 × 32 pixels for experiments in this subsection.  Figure 5 shows sample images of one person.

#### 4.2.1. Parameter Selection

Feature extraction methods need to select insensitive parameters [39]. We need to tune three parameters, that is, *λ*, *μc*, and *ρ*, for SMEDP. So, an experiment on parameter sensitivity is conducted in this subsection. Since it is difficult to tune the three parameters simultaneously, the strategy of grid search [39] is employed to select the parameter. The core idea of grid search is fixing one parameter and tuning the others. Specifically, 8 images per class are randomly selected in the ORL database for training and the remaining for testing. The number of principal components is set to 290 during the PCA step. Then, we perform SMEDP to convert the 290-dimensional representation to a 110-dimensional map. Finally, we use the NN classifier with cosine distance for classification. The experiment is run 50 times, and the results are reported in Figure 6.

Two cases are used to evaluate the effects of different parameter settings: (1) Fix *ρ* = 1.1, tune *λ* and *μc* from {0.0001, 0.001, 0.01, 0.1, 1}.  Figure 6(a) shows the results, and it is obvious that the parameter *λ* and *μc* do affect the performance of SMEDP. When *λ* = 0.01, 0.1, 1 and *μc* = 0.01, 0.001, 0.0001, the performance of SMEDP changes a little and the recognition rate is more than 90%. When *λ* = 0.1 and *μc* = 0.01, SMEDP achieves the best effect; (2) fix *λ* = 0.1 and *μc* = 0.01, vary *ρ* from {0.1, 0.15, 0.2, 0.25, 0.3, 0.35, 0.4, 0.45, 0.5, 0.55, 0.6, 0.65, 0.7, 0.75, 0.8, 0.85, 0.9, 0.95, 1.0, 1.05, 1.1, 1.15, 1.2, 1.3, 1.35, 1.4, 1.45, 1.5, 1.55}.  Figure 6(b) gives the average recognition rate curves of SMEDP with different values of *ρ*. From Figure 6(b), we can find that SMEDP is robust with different *ρ*, which means parameter *ρ* has a certain degree of influence on the recognition rate, but the influence is insignificancy. To facilitate the analysis of data, the part of Figure 6(b), where the recognition rate ranges from 87% to 93%, is shown in Figure 6(c). Besides, from the results, we can find that *ρ* with a value of 1.1 produces better performance. Overall, the above analysis provides a guidance of parameters selection for SMEDP in follow-up experiments.

The article "A Smoothed Matrix Multivariate Elliptical Distribution-Based Projection Method for Feature Extraction" was published in 2022. Journal: Comput Intell Neurosci.

#### 4.2.2. Classification Results with Different Expressions and Illuminations

We construct classification experiments to evaluate the robustness of SMEDP with different expressions and illuminations. We also compare SMEDP with PCA, LPP, SPP, CRP, and NMRP. The parameters of each method are set as follows: (1) nearest neighbor point *k* in LPP is set to 20; (2) Justin Romberg's l1qc_logbarrier is used to calculate L1-norm and *λ* is set to 1e-3 in SPP; (3) in CRP and NMRP, *λ* is set to 0.1 and 1, respectively; (4) for SMEDP, the parameters *λ*, *μc*, and *ρ* are set as 0.1, 0.01, and 1.1, respectively. We run the experiments 50 times. In each run, *l* (= 5, 6, 7, and 8) images are randomly selected from each subject as a training set and the rest 10-*l* images are treated as a test set. Besides, SPP, CRP, NMRP, and SMEDP all apply a PCA preprocess step to reduce the dimensions of the raw data. For *l* (=5, 6, 7, and 8), the numbers of principal components are set to 170, 210, 250, and 290, respectively. Finally, the numbers of subspace dimensions by all the methods except SPP are varied from 50 to the numbers of principal components at intervals of 30, 40, 50, and 60. Since SPP is sensitive to large variations in pose, the numbers of subspace dimensions for ORL database are varied from 30 to 50 to maintain a relatively high level of recognition rate.  Figure 7 shows the average recognition results of different methods, and Table 1 (the best performing method has been highlighted) gives the average maximal recognition rate of each method.

From the results, we can see that SMEDP performs the best, which verifies that it can preserve the primary discriminant information for classification. Specifically, SMEDP can outperform the others by about 2% improvement on *l* (= 5, 6) and about 1% improvement on *l* (= 7, 8). Since NMRP and SMEDP get an adjacent weight matrix by matrix regression, their results are closer. Moreover, CRP, which is based on vector regression, achieves a performance comparable to NMRP in most cases. This is mainly because collaborative representation can improve the discriminating capability to some extent. Since the limitations of PCA, LPP, and SPP mentioned above, the classification performance of them is poor.

The article "A Smoothed Matrix Multivariate Elliptical Distribution-Based Projection Method for Feature Extraction" was published in 2022. Journal: Comput Intell Neurosci.

### 4.3. Experiments on CMU PIE Face Database

CMU PIE face database [40] consists 41,368 images of 68 people. All images are taken from different poses, illumination, and facial expressions for each individual. We choose C09 (one of five subsets of near frontal poses, which contains 1632 images) for the test. All images were in grayscale and resized to 64 × 64 pixels.  Figure 8 shows sample images of one person.

#### 4.3.1. Classification Results with Different Illuminations

For evaluating the robustness of SMEDP to the data with different illuminations, we conduct experiments and systematically compare it with the methods mentioned in Section 4.2.2. Specifically, we choose the first *l* (=7, 9, 11, 13) images of one person for training and the rest 24-*l* images for testing. It is worth noting that LPP, SPP, CRP, NMRP, and SMEDP all involve the selection of parameters, and they are adjusted based on grid search. In this subsection, they are set as follows: (1) nearest neighbor point *k* in LPP is set to 20; (2) in SPP, Justin Romberg's l1qc_logbarrier is used to calculate L1-norm and *λ* is set to 1e−4; (3) in CRP and NMRP, *λ* is set to 0.01 and 0.1, respectively; (4) for SMEDP, *λ*, *μc*, and *ρ* are set as 0.01, 0.01, and 1.1, respectively. PCA is first used to preprocess the images. We set the dimensions of the PCA subspace to 300, 250, 200, and 150, which correspond to *l* (=7, 9, 11, 13), respectively.  Figure 9, Tables 2 and 3 show the results. Note that numbers in bold mean the best results in Tables 2 and 3.

From the experimental results, it can be seen that the recognition rate of these methods generally increases with the growth of the feature dimensions. Our proposed SMEDP always obtains the best results, which demonstrates its robustness to illumination variations. One can also note that SMEDP can outperform the others by about 2% improvements on 150 dimensions when *l* = 7 and 11. Besides, NMRP and CRP are comparable to SMEDP in some cases since the former takes advantage of matrix structure and the latter uses collaborative representation to preserve the primary discriminant information. SPP is superior to PCA and LPP, but inferior to SMEDP and NMRP. The superiority is distinctive because the sparsity properties are considered in the construction of graph. PCA and LPP perform worse than others. The reason is that they only take global structure or local structure of data into account.

The article "A Smoothed Matrix Multivariate Elliptical Distribution-Based Projection Method for Feature Extraction" was published in 2022. Journal: Comput Intell Neurosci.

#### 4.3.2. Classification Results with Block Occlusions

In this subsection, we verify the robustness of SMEDP. We use the similar experiment setting as in Section 4.3.1. First 13 samples are selected as a training set and the rest samples with random occlusions of black blocks or white blocks are treated as a test set. The block size determines the occlusion level of an image. We use PCA to reduce the dimension of data to 150, and then, classification tests were carried out on the test samples with varying degrees of random occlusions.  Figure 10 shows the results.

From Figure 10, it is evident that the recognition rates of PCA and LPP are low whether the samples under the occlusions of black blocks or white blocks. It means that they cannot handle the structural noise very well. The proposed SMEDP is superior to some SR-based feature extract methods (SPP and CRP). But the performance of NMRP is very close to SMEDP when the occlusion level is no more than 30%, that is, because they are all based on matrix regression, which can get more discriminative information from corrupted data. As the level of occlusion rises, NMRP no longer has an advantage, and the smoothed matrix multivariate elliptical distribution plays a role in SMEDP. Overall, this experiment confirms SMEDP is more robust than the others with block occlusions.

## 5. Conclusions

A method called smoothed matrix multivariate elliptical distribution-based projections (SMEDP) is proposed in this paper. Specifically, we use a modified SMED to automatically construct an adjacency graph and then learn an optimal projection matrix in the PCA subspace. Since SMED considers both the global structure and the local structure based on sparse and low-rank representation, SMEDP can get more discriminative information from corrupted data. Experimental results on three databases show that SMEDP achieves considerable visual and recognition performance. Specifically, its robustness to illumination variations and block occlusions.

However, each method has its own strengths and weaknesses. SMEDP separates graph embedding and projection learning into two independent processes, which makes it difficult to learn the optimal projection matrix once the graph embedding is invalid. Furthermore, although SMEDP contains the natural discriminating information, it ignores the label information of the data, which will still affect the discriminative ability of the model. In the future, we will consider to simultaneously perform graph embedding and projection learning in a unified objective function and introduce the class label information in graph construction to extend SMEDP to the supervised scenario. We believe that the improvement of SMEDP will have better performance for pattern recognition task.

The article "A Smoothed Matrix Multivariate Elliptical Distribution-Based Projection Method for Feature Extraction" was published in 2022. Journal: Comput Intell Neurosci.

## Figures and Tables

**Figure 1:** The flowchart of SMEDP. Given some sequential data, SMEDP utilizes a modified SMED to automatically build the graph.

**Figure 2:** Some images from COIL-20.

**Figure 3:** Images of 10 objects from COIL-20.

**Figure 4:** Visualizations of 50 images on COIL-20. (a) PCA. (b) LLE. (c) ISOMAP. (d) LPP. (e) SPP. (f) CRP. (g) NMRP. (h) SMEDP.

**Figure 5:** Sample images of one person from ORL.

**Figure 6:** The classification performance of SMEDP for varying values of *λ*, *μc*, and *ρ* on ORL. (a) The average recognition rate of SMEDP with different values of *λ* and *μc*. (b) The average recognition rate curves of SMEDP with varying values of *ρ*. (c) The part of Figure 6(b) where the recognition rate ranges from 87% to 93%.

**Figure 7:** Recognition rate (%) versus subspace dimension on ORL. (a) *l* = 5. (b) *l* = 6. (c) *l* = 7. (d) *l* = 8.

**Figure 8:** Sample images of one person from CMU PIE.

**Figure 9:** Recognition rate (%) versus subspace dimension on CMU PIE. (a) *l* = 7. (b) *l* = 9. (c) *l* = 11. (d) *l* = 13.

**Figure 10:** Recognition rate (%) under the different occlusion levels on CMU PIE. (a) The occlusion of black block. (b) The occlusion of white block.

**Algorithm 1:** Iterative Algorithm for solving *α*.

**Algorithm 2:** SMEDP.

**Table 1:** Average recognition rate (%) and standard deviation of different methods on ORL.

Methods	*l* = 5	*l* = 6	*l* = 7	*l* = 8
PCA	0.7466 ± 0.03254	0.7886 ± 0.02666	0.8245 ± 0.02511	0.8593 ± 0.03828
LPP	0.7455 ± 0.02937	0.7876 ± 0.03026	0.8233 ± 0.02761	0.8563 ± 0.03456
SPP	0.7265 ± 0.03429	0.7806 ± 0.03386	0.8315 ± 0.03525	0.8643 ± 0.03805
CRP	0.8230 ± 0.02229	0.8658 ± 0.02426	0.8950 ± 0.02630	0.9140 ± 0.02797
NMRP	0.8185 ± 0.02423	0.8595 ± 0.02735	0.8975 ± 0.02860	0.9170 ± 0.02597
SMEDP	**0.8427** ± 0.02548	**0.8776** ± 0.02273	**0.9073** ± 0.02671	**0.9253** ± 0.02521

**Table 2:** Recognition rates (%) and versus subspace dimension of different methods on CMU PIE with *l* = 7, 9.

Methods	*l* = 7					*l* = 9				
	*d* = 30	60	90	120	150	*d* = 30	60	90	120	150
PCA	0.2180	0.2647	0.2673	0.2829	0.2846	0.3127	0.3755	0.4137	0.4275	0.4324
LPP	0.2266	0.2604	0.2768	0.2785	0.2898	0.2971	0.3912	0.4265	0.4422	0.4637
SPP	0.1254	0.1877	0.2569	0.3365	0.3538	0.3618	0.5078	0.6559	0.7539	0.8265
CRP	0.2820	**0.3867**	0.4602	0.5398	0.6151	0.4598	0.6013	0.7127	0.7745	0.8216
NMRP	0.2197	0.3175	0.4394	0.5311	0.6073	0.4598	0.6078	0.7363	0.8020	0.8510
SMEDP	**0.2967**	0.3824	**0.4810**	**0.5631**	**0.6324**	**0.4759**	**0.6294**	**0.7369**	**0.8122**	**0.8571**

The article "A Smoothed Matrix Multivariate Elliptical Distribution-Based Projection Method for Feature Extraction" was published in 2022. Journal: Comput Intell Neurosci.

**Table 3:** Recognition rate (%) and versus subspace dimension of different methods on CMU PIE with *l* = 11, 13.

Methods	*l* = 11					*l* = 13				
	*d* = 30	60	90	120	150	*d* = 30	60	90	120	150
PCA	0.3127	0.3755	0.4138	0.4275	0.4326	0.4920	0.4973	0.5321	0.5348	0.5321
LPP	0.2971	0.3912	0.4265	0.4422	0.4637	0.4612	0.5749	0.6150	0.6056	0.6310
SPP	0.3618	0.5078	0.6559	0.7529	0.8265	0.6484	0.8396	0.8997	0.9559	0.9679
CRP	**0.5098**	**0.6333**	0.7127	0.7745	0.8216	0.7233	0.8670	0.9225	0.9372	0.9599
NMRP	0.4598	0.6078	**0.7363**	0.8020	0.8510	0.7219	0.8610	**0.9345**	**0.9679**	0.9733
SMEDP	0.4059	0.5794	0.7069	**0.8022**	**0.8571**	**0.7286**	**0.8636**	0.9305	0.9626	**0.9779**

## Data Availability

The dataset can be accessed upon request (https://www.cad.zju.edu.cn/home/dengcai/Data/FaceData.html).
